This article has been retracted.

# Dexmedetomidine Regulates the miR-146a-5p/NF-*κ*B Axis to Alleviate Electroconvulsive Therapy-Induced Cognitive Impairments

**DOI:** 10.1155/2022/8371492

**Published:** 2022-10-04

**Authors:** Xiaohui Zhou, Peipei Si, Li Wang, Huiqun Jia

**Affiliations:** ^1^Department of Anesthesiology, The First Hospital of Hebei Medical University, Shijiazhuang, Hebei, China; ^2^Department of Neurology, The Second Hospital of Hebei Medical University, Shijiazhuang, Hebei, China; ^3^Department of Anesthesiology, The Fourth Hospital of Hebei Medical University, Shijiazhuang, Hebei, China

## Abstract

Electroconvulsive therapy (ECT) is a nonpharmacological treatment for depressive episodes and other psychiatric disorders. It is used to control the condition by causing a transient loss of consciousness through electrical stimulation. Dexmedetomidine (DEX) is a novel and highly selective adrenergic agonist with sedative, sympathetic nerve activity inhibiting and stress-responsive effects. This study focused on the effect of DEX on cerebral protection after ECT treatment. 68 depression patients were enrolled and divided into control group and DEX group. The occurrence of delirium after ECT treatment in depression cases was recorded. In vivo, we constructed chronic mild and unpredictable stress (CUMS) rats to mimic depression model. Meanwhile, ECT treatment and DEX injection were administrated in CUMS rats. Learning and memory in rats were measured by Morris water maze test, open field test (OFT), and forced swimming test (FST). Finally, the expression of miR-146a-5p and NF-*κ*B was determined by RT-qPCR and western blot assay. The incidence of delirium after ECT treatment was prominently reduced in DEX group in relation to control group. In vivo, DEX injection had no effect on ECT treatment efficacy against depression conditions. After ECT treatment, the cognitive impairment was ameliorated in CUMS rats accomplished with decreased miR-146a-5p and increased NF-*κ*B level. Finally, compared with ECT treatment, DEX injection could protect against depression-like behaviors by increasing miR-146a-5p level and inactivated NF-*κ*B pathway. Overall, ECT-induced cognitive impairment in depression rats could be ameliorated by DEX injection via miR-146a-5p/NF-*κ*B axis.

## 1. Introduction

The main clinical manifestations of depression are symptoms that slowed thinking and reduced volitional activity, which may be accompanied by somatic symptoms, suicidal ideation, and behavior [1]. As a very common mental illness, depression is the third leading cause of disability in the world [2]. Depression's processing bias of emotional information is associated with recovery from impaired mood, in part by promoting persistent negative mood to maintain a depressed state [3]. In addition to manifesting processing biases to emotional information, depression also manifests as a lack of pleasure, and often clinically as reduced motivational drive and satisfaction [4]. The clinical manifestations of depression are diverse, but its mechanisms remain unclear.

Chronic unpredictable mild stress (CUMS) has been extensively used as a mechanism to induce depression-like behaviors in experimental animals to examine the pathophysiology of depression [5]. CUMS models are often related to increased anxiety-like behaviors and impaired hypothalamic-pituitary-adrenocortical (HPA) axis function. CUMS models are linked to decreased sucrose intake and decreased reactivity, which are the main symptoms of anhedonia, a major feature of depression [6].

Electroconvulsive therapy (ECT) is one of the most effective treatment options for depressed patients who do not respond to psychotropic medication or psychotherapy and is primarily used to support the treatment of major depression, especially in patients with severe illness symptoms [7–9]. ECT mainly involves stimulating the cortical cells with a certain electric current to produce widespread spontaneous discharges, causing the patient to experience generalized convulsion symptoms [5, 7]. Studies have shown that ECT is reliable for the treatment of psychiatric disorders, but it can affect the cognitive function of patients to a certain extent, leading to symptoms of cognitive impairment, which limits its clinical application value to a certain extent [10]. Many of the negative views can be traced back to the early days of ECT, when it was administered without muscle relaxants and anesthesia [11]. For instance, clinical practice has shown that ECT treatment may cause slight damage to the brain tissue and nervous system of patients, resulting in short-term memory impairment [12, 13]. In the last decade, improvements in the way ECT is performed, such as the use of anesthetic drugs, have significantly improved the safety of ECT [14, 15]. Therefore, it is important to strengthen the brain protection during ECT treatment.

In recent years, ECT combined with anesthetic drugs has been modified from traditional ECT treatment, and the use of modified medication has been reported to help improve patient treatment tolerance and safety [14, 15]. Among common anesthetic drugs, dexmedetomidine (DEX), a highly selective *α*2 agonist with sedative, anti-inflammatory and antisympathetic effects, improves cognitive function in rats by reducing inflammatory responses in the central nervous system [16–18].

Nuclear factor kappa B (NF-*κ*B) is a crucial transcription factor that influences chronic diseases by promoting inflammatory responses [16]. Activation of the NF-*κ*B has been reported to be closely related to cognitive impairments [17]. p65 is considered as the main activator within NF-*κ*B. NF-*κ*B can be activated by A*β*, leading to phosphorylation of its p65 subunit and transfer to the nucleus, thus enhancing the transcription of proinflammatory cytokines [18].

MicroRNAs (miRNAs) are a family of short, single-stranded noncoding RNAs that play a crucial role in suppressing target gene expression through mRNA degradation or translational inhibition [19]. miRNAs take part in the development of postoperative cognitive dysfunction in the central nervous system and neuropsychiatric diseases, such as ischemic stroke and Alzheimer's disease [20].

In this study, we aimed to study whether DEX injection could mitigate cognitive impairment and cerebral injury under depression conditions after ECT treatment. To this end, we recruited depression patients and constructed depression rats in vivo. The influence of DEX on ECT treatment was measured accordingly.

## 2. Materials and Methods

### 2.1. Patients Enrollment

68 depression patients admitted to the First Hospital of Hebei Medical University from May 2019 to January 2021 were selected as subjects including 29 males and 39 females (aged 19-58 years old). Inclusion criteria: (1) meeting the diagnostic criteria of WHO International Classification of Diseases Manual and Chinese Classification and Diagnostic Standard of Mental Disorders; (2) Brief Psychiatric Rating Scale (BPRS) score ≥ 35 and Positive and Negative Symptom Scale (PANSS) score ≥ 60; (3) poor effect of medication, with impulsivity, hallucinations, and delusions. Exclusion criteria: (1) patients with severe respiratory, cardiovascular, and cerebrovascular system diseases and infectious diseases associated with inflammatory reactions; (2) uncontrollable behavioral disorders and schizoaffective psychosis; (3) patients with psychotic disorders caused by psychoactive and nonaddictive substances, organic psychiatric disorders, and other diseases with concomitant psychosis. The study was approved by the Ethics Committee of the First Hospital of Hebei Medical University, and informed consent was signed with the patients and their families.

All enrolled patients were randomly divided into two groups: DEX group, injection with 1.0 *μ*g/kg DEX and control group, injection with corresponding volume of saline. Each patient was given intravenous atropine 0.5 mg before dosing. The DEX group was injected with DEX (batch number: H20090248, Jiangsu Hengrui Pharmaceutical Co., Ltd.). Briefly, 200 *μ*g of DEX was diluted to 50 ml with saline and prepared to a concentration of 4 *μ*g/ml. Meanwhile, the control group was injected with the corresponding volume of saline. After the injection, propofol and succinylcholine were administered to induce intravenous anesthesia. After the anesthesia took effect, 6 ECTs were performed with an ECT device (SOMATICS, LLC, USA). In brief, a psychiatrist authorized to operate ECT techniques stimulated the patients' temporal region bilaterally with an energization time of 2 to 4 s; effective treatment was considered when the patient exhibited spasticity in the muscles of the face, eyes, and extremities. Treatment was given every other day for a total of 6 sessions for 2 weeks.

### 2.2. Assessment Criteria

The occurrence of delirium after ECT was observed, and the level of CRP concentration before and after ECT was also measured in each group. Briefly, 5 m L of fasting venous blood was drawn from each subject before and after treatment. Then, the sample was collected after centrifugation (3000 r/min,10 min), and the CRP level was measured by immunoprojection turbidimetry. The incidence of delirium was evaluated using the Richmond Agitation Sedation Scale (RASS) and the delirium assessment method, the Confusion Assessment Method (CAM).

### 2.3. Animal Experiment

60 female SD rats (5 weeks old, weighing 140-160 g) from the First Hospital of Hebei Medical University were acclimatized for 1 week. Rats were housed under standard conditions (12/12 h of dark/light, 55 ± 10%relative humidity, and 23 ± 2°C room temperature). All animal protocols were approved by the Animal Ethics Committee of the First Hospital of Hebei Medical University and were performed in accordance with the National Institutes of Health Guide for the Care and Use of Laboratory Animals. In accordance with international guidelines, every effort was made to minimize animal suffering. Chronic mild and unpredictable stress (CUMS) rats received 1 of the following 5 stressors per day: wet bedding for 24 h; behavioral restraint for 24 h; cage tilted at 45° for 24 h; water or food fasting for 24 h; swimming in ice water at 4°C or hot water at 42°C for 5 min. The same stimuli were not applied, and the experiment was conducted consecutively for 22 days.

### 2.4. ECT Treatment

After the depression model was successfully established, CUMS rats were randomly divided into CUMS group, ECT group, ECT + DEX group, ECT + DEX + antagomiR-NC group, and ECT + DEX + antagomiR-146a-5p group, with the number of 12 rats in each group. ECT rats were treated with YSD-4G ECT machine once a day for 7 days. DEX rats were given DEX injection 25 *μ*g/kg intraperitoneally.

The miR-146a-5p antagonist (antagomiR-146a-5p) and its negative control (antagomiR-NC) were synthesized by Shanghai GenePharma. 20 nmol of antagomiR-146a-5p and antagomiR-NC were injected into the rats once every other day for three times. The miR-146a-5p antagonist in this experiment was antagomiR-146a-5p, which was specially chemically modified to have high stability and inhibit the function of miRNA in animals in vitro and in vivo.

### 2.5. Sucrose Preference Test (SPT)

Before the first test, all rats were trained to acclimate to a 1% sucrose solution (w/v) in a quiet environment. Two bottles of 1% sucrose solution were placed on each cage for 24 h, and then one bottle of 1% sucrose solution was replaced with pure water for 24 h. After acclimation, the rats were deprived of food and water for 24 h. SPT was performed the next morning, and the rats were fed two bottles of preweighed liquid meanwhile: one containing 1% sucrose solution and one pure water. The bottles were balanced on the left and right sides of the cage throughout the experiment to avoid positional preference effects. 8 h later, the consumption of sucrose water and tap water was measured. Sucrose preference (%) = sugar − water consumption/(sugar − water consumption + tap water consumption) × 100%.

### 2.6. Morris Water Maze Test

The Morris water maze test consisted of a training experiment and a test experiment to investigate the learning and memory abilities of the objects [21].

Training experiment: 7 d before the modeling, the rats were put into the water facing the wall of the pool and were free to find the platform (2 cm above the water surface); if they did not find it within 5 min, they were pulled to the platform and stayed for 10 s to let them remember, and then put back into the cage. Test experiment: The rats were placed in the water from the direction facing the wall of the pool, and the latency time of climbing onto the platform was recorded within 30 s. The target quadrant memory time of the rat was recorded by removing the platform and recording the time spent in the quadrant where the original platform was located within 90 s.

### 2.7. Open Field Test (OFT)

The OFT test is used to assess the motor activity and emotional response of objects. The device is a 120 cm × 90 cm × 35 cm opaque open box [22]. The perimeter is black, and the bottom is divided into 25 squares by white lines. The outer 16 squares are considered the peripheral field, and the middle 9 squares are considered the central area. In a quiet environment, each rat was placed individually in a corner of the apparatus and allowed to explore freely for 5 min. The rats were placed in the laboratory 30 min before the test to acclimatize to the environment. After each test, the apparatus was thoroughly cleaned with 70% ethanol. Rats were analyzed by behavioral video for distance traveled in the central zone and time spent in the central zone.

### 2.8. Forced Swimming Test (FST)

Forced swimming system (Etho Vision XT) was used for the experiment. Rats were forced to swim in a vertical plastic cylinder (30 cm in diameter and 50 cm in height) with 30 cm of water in the container, held at 25°C. All rats were placed one by one in the water for 15 min, then dried and returned to the cage. 24 h later, the rats were placed again one by one in the water, and each rat was recorded by video camera for 5 min. The water was replaced after each trial. The immobility time during this period was recorded. The immobility was quantified as the time when the rats floated in the water without struggling and only had the necessary movements to keep their heads above the water surface or touch the bottom of the pool for more than 1 s.

### 2.9. RT-qPCR Analysis

Total RNA was extracted from rat hypothalamic tissue by Trizol reagent, and the concentration and purity were determined by NanoDrop. 2 *μ*g of total RNA was extracted, and cDNA was obtained by reverse transcription using Promega M-MLV reverse transcription kit. cDNA was amplified by PCR, and miR-146a-5p was detected by ALL-in-One miRNA RT-qPCR Detection Kit, with U6 as the internal reference. Amplification was performed at 50°C for 20 min, followed by 95°C for 15 min and 45 cycles at 95°C for 10 s. The relative expression of miR-146a-5p was measured by the 2^−ΔΔCT^ method. The primer sequences were listed as follows: miR-146a-5p forward, 5′-CCGATGTGTATCCTCAGCTTTG-3′ and reverse, 5′-GCCTGAGACTCTGCCTTCTG-3′; U6 forward, 5′-ATTGGAACGATACAGAGAAGATTAG-3′ and reverse, 5′-TGCGTGTCGTGGAGTC-3′.

### 2.10. Western Blot Assay

The rat hypothalamus tissues were lysed by RIPA method, and the total protein was collected by centrifugation at 12000 r/min for 10 min. About 50 *μ*g sample was taken for electrophoresis using 10% SDS-PAGE and transferred to a PVDF membrane. Then, the membranes were placed in 5% skimmed for blocking. After blocking, the membranes were incubated overnight at 4°C with primary antibodies p-NF-*κ*B (ab288751, 1 : 1000), NF-*κ*B (ab210924, 1 : 1000), and GAPDH (ab8245, 1 : 1000). On the second day, the membranes were incubated at room temperature for 1 h with secondary antibody H&L (DyLight^®^ 488) (ab96879, 1 : 1000). Finally, high-sensitivity chemiluminescent reagents were added for color development. Gel image analysis was performed using Image J software, and the relative expression of the protein was calculated using GAPDH as the internal reference. All antibodies were obtained from Abcam (Shanghai, China).

### 2.11. Statistical Analysis

SPSS18.0 and GraphPad 7.0 software were used for statistical processing. Three independent experiments were carried out in this study. The data were tested for normality and chi-squaredness. The measurement data conforming to normal distribution were expressed as mean ± standard deviation (SD). Student's *t*-test was used for comparison between two means while one-way ANOVA was used for comparison between multiple groups. The difference was statistically significant at *P* < 0.05.

## 3. Results

### 3.1. Basic Information of All Enrolled Depression Patients

The demographic and clinicopathological information of all 68 enrolled depression patients are shown in Table 1. As shown in Table 1, there were no significant differences in gender, age, body weight, BRPS score, and PANSS score between control group and DEX group (*P* > 0.05).

### 3.2. The Occurrence of Delirium of Enrolled Patients

The incidence of delirium in two groups after 6 times of ECT was recorded in Table 2. As depicted in Table 2, the incidence of delirium was dramatically decreased in DEX group as compared with control group.

### 3.3. DEX Had No Effect on ECT against Depression-like Behaviors

As to confirm whether DEX had effect on ECT treatment, we performed SPF test. As shown in Figure 1, compared with sham group, CUMS rats had unfavorable SPF percentage (*P* < 0/05), implying the success of depression rats modeling. Moreover, after ECT treatment, the SPF percentage was better than CUMS groups (*P* < 0.05). However, there were no significant differences between ECT and ECT + DEX group (*P* > 0.05). The above results suggested that DEX injection had no effect on ECT against depression-like behaviors.

### 3.4. DEX Mitigated ECT-Induced Cognitive Impairment in Depression Rats by Upregulating miR-146a-5p and Inactivating NF-*κ*B Pathway

As to confirm the effect of DEX on cerebral protection after ECT treatment under depression conditions, we constructed Morris maze test, OFT test, FST test, RT-qPCR assay, and western blot analysis. First, the results in Figures 2–5 demonstrated that CUMS rats were successfully built compared with sham group (*P* < 0.05, *P* < 0.01, and *P* < 0.001). Moreover, after ECT treatment, the escape latency and immobility time were hindered, while platform crossing number, percentage target quadrant time, and central distance were enhanced (*P* < 0.05, *P* < 0.01, and *P* < 0.001), suggesting that ECT treatment could ameliorate cognitive impairment in depression rats. Furthermore, the escape latency and immobility time were decreased, while platform crossing number, percentage target quadrant time, and central distance were increased in ECT + DEX group in relation to ECT group (Figures 2–4, (*P* < 0.05, *P* < 0.01, and *P* < 0.001)). However, the change induced by DEX injection could be partially counteracted by antagomiR-146a-5p injection. Finally, as depicted in Figures 5 and 6, in relation to sham rats, CUMS rats presented NF-*κ*B signaling activation and decreased miR-146a-5p level (*P* < 0.05 and *P* < 0.01); moreover, ECT treatment enhanced the activation or decrease further ((*P* < 0.05 and *P* < 0.01). Compared with ECT group, combination with DEX injection could increase miR-146a-5p level while inactivate NF-*κ*B pathway (*P* < 0.01 and *P* < 0.001). Moreover, the inactivation of NF-*κ*B pathway could be rescued by injection with antagomiR-146a-5p.

## 4. Discussion

ECT is more effective in treating psychiatric disorders, including depression [23, 24]. However, the mechanisms by which ECT induced the onset of psychiatric symptoms such as delirium in patients have not been fully elucidated to date [25]. Delirium is a common adverse effect of ECT after long-term application in depressed patients [26]. Up to date, the application of anesthetic drugs is an important breakthrough in the shackles of ECT treatment. In our experiment, we used CUMS rats to construct depression in vivo model. As shown, CUMS rats presented unfavorable sucrose preference, impaired cognitive function, implying that the depression-like rats were successfully built.

With the rapid development of medical technology, the combination of advanced anesthesia techniques with ECT has greatly reduced the harm to patients during treatment [26]. The commonly used anesthetic drugs in clinical practice are propofol, ketamine, etomidate, and DEX [27–30]. DEX is a highly selective *α*2-adrenergic agonist with sedative and analgesic effects and no adverse effects on the patient's respiratory and circulatory systems. Previous studies have found that DEX has the effect of preventing the occurrence of delirium during the implementation of ECT [25, 31, 32]. More importantly, DEX has been reported to prevent of postoperative delirium and cognitive dysfunction [33]. Consistent with previous study, our study demonstrated that DEX injection could reduce the incidence of delirium during ECT treatment. Moreover, in vivo experiments further revealed that DEX injection depression rats could ameliorate ECT-induced memory and learning impairment, thereby improving cerebral injury. However, the specific molecule by which DEX improved ECT-induced cerebral impairment remained obscure.

Accumulating evidence suggested that DEX participated in protecting brain injury by regulating various miRNAs expressions. For instance, Li et al. reported that DEX could downregulate miR-27a-3p level to deplete inflammation and autophagy in traumatic brain injury [34]. Guan et al. and He et al. uncovered that miR-134a-5p and miR-20a-5p expressions were depleted by DEX, thereby alleviate hypoxia-ischemic brain injury [35, 36]. Another research found that DEX could enhance miR-429-3p level which may contribute to attenuate cognitive impairment caused by cisplatin [37]. As was a widely reported miRNA, miR-146a-p was unveiled to participate in regulating depression development. For instance, Li et al. [34] elucidated that enhanced miR-146a-5p by exosomes could inhibit neurogenesis, thereby alleviating depression process. Guan et al. [35] illustrated that miR-146a-5p might be a feasible antidepressant factor. In this study, we discovered that DEX could increase miR-146a-5p level during ECT treatment, which were in concordance with previous studies [38, 39].

Previous studies have confirmed that miR-146a-5p could inactivate or suppress NF-*κ*B pathway [38, 39]. NF-*κ*B is an important transcription factor that regulates immune inflammation-related genes, and when high expression of NF-*κ*B p65 was induced, it could in turn trigger the inflammatory response. According to several researches, NF-*κ*B pathway was activated in depression. Meanwhile, usage of DEX could hinder NF-*κ*B activation as well. Consistently, rescue experiments in our study verified that DEX could mitigate ECT-induced memory and learning impairment in depression rats by increasing miR-146a-5p level and inactivating NF-*κ*B pathway.

There are several limitations in our study. First, the specific mechanism of CET on regulating the NF-*κ*B pathway was not investigated. Second, the target mRNAs of miR-146a-5p were not investigated. In addition, the samples of our study were relatively small. Therefore, our study should perform more relevant experiments to perfect our study.

In summary, we found that DEX alleviated ECT-induced cognitive impairment in depressed rats but did not alter the antidepressant effect of ECT. The potential neuroprotective mechanism of DEX may be reached by increasing the expression of miR-146a-5p and inhibiting the activation of NF-*κ*B signaling pathway.

## Figures and Tables

**Figure 1:** Sucrose preference percentage in different groups. ^∗∗^*P* < 0.01, CUMS vs. sham group; ^##^*P* < 0.01, ECT vs. CUMS group.

**Figure 2:** Morris water maze test. (a) Escape latency result. (b) Platform crossing number. (c) Percentage of target quadrant time. ^∗^*P* < 0.05, ^∗∗^*P* < 0.01, CUMS vs. sham group; ^#^*P* < 0.05, ^###^*P* < 0.001, ECT vs. CUMS group; ^&&^*P* < 0.01, ^&&&^*P* < 0.001, ECT + DEX vs. ECT group; ^+^*P* < 0.05, ^+++^*P* < 0.001, ECT + DEX + antagomiR-146a-5p vs. ECT + DEX + antagomiR-NC group.

**Figure 3:** OFT test. Central distance was recorded in OFT test. ^∗∗^*P* < 0.01, CUMS vs. sham group; ^###^*P* < 0.001, ECT vs. CUMS group; ^&^*P* < 0.05, ECT + DEX vs. ECT group; ^+^*P* < 0.05, ECT + DEX + antagomiR-146a-5p vs. ECT + DEX + antagomiR-NC group.

**Figure 4:** FST test. Immobility time was recorded in FST test. ^∗∗∗^*P* < 0.001, CUMS vs. sham group; ^##^*P* < 0.01, ECT vs. CUMS group; ^&&&^*P* < 0.001, ECT + DEX vs. ECT group; ^++^*P* < 0.01, ECT + DEX + antagomiR-146a-5p vs. ECT + DEX + antagomiR-NC group.

**Figure 5:** RT-qPCR result measured miR-146a-5p in rat hypothalamic tissues. ^∗^*P* < 0.05, CUMS vs. sham group; ^##^*P* < 0.01, ECT vs. CUMS group; ^&&&^*P* < 0.001, ECT + DEX vs. ECT group; ^++^*P* < 0.01, ECT + DEX + antagomiR-146a-5p vs. ECT + DEX + antagomiR-NC group.

**Figure 6:** Western blot assay detected NF-*κ*B pathway in rat hypothalamic tissues. ^∗∗^*P* < 0.01, CUMS vs. sham group; ^#^P < 0.05, ECT vs. CUMS group; ^&&^*P* < 0.01, ECT + DEX vs. ECT group; ^++^*P* < 0.01, ECT + DEX + antagomiR-146a-5p vs. ECT + DEX + antagomiR-NC group.

**Table 1:** Basic information of all enrolled subjects.

	Control group (*n* = 34)	DEX group (*n* = 34)	*P* value
Gender			0.3268
Male	17	12	
Female	17	22	
Age (years)	33.5 ± 5.4	35.7 ± 6.1	0.1201
Body weight	61.5 ± 7.2	62.9 ± 8.8	0.4320
BRPS score	39.5 ± 2.4	40.2 ± 3.2	0.3113
PANSS score	69.2 ± 2.3	68.6 ± 2.4	0.2964

**Table 2:** The occurrence of delirium after ECT in two groups.

Grouping	1^st^ ECT	2^nd^ ECT	3^rd^ ECT	4^th^ ECT	5^th^ ECT	6^th^ ECT	Total incidence (%)
Control group (*n* = 34)	8	11	11	7	12	5	26.47% (54/204)
DEX group (*n* = 34)	5	6	4	3	5	2	12.25% (25/204)

## Data Availability

Original data are available from the corresponding author under reasonable requests.
